# Application Research of Humanistic Care and Situational Integration in Nursing of Schizophrenia in Recovery Period

**DOI:** 10.1155/2022/4705107

**Published:** 2022-09-22

**Authors:** Yanhua Zhang

**Affiliations:** Rehabilitation Department, Hangzhou Fuyang Third People's Hospital, Hangzhou 311400, Zhejiang, China

## Abstract

**Objective:**

To formulate corresponding nursing humanistic care measures according to the needs of patients, evaluate the intervention effect of patients, and provide reference for nursing staff to better provide nursing humanistic care for patients with schizophrenia in convalescence.

**Methods:**

Using the random number table method, 110 inpatients with convalescent schizophrenia were randomly divided into the control group (*n* = 55) and the experimental group (*n* = 55). The sample *t*-test was used to compare the changes of patient insight, treatment attitude, rehabilitation efficacy, and negative emotion score before and after nursing humanistic nursing intervention, and analyze the effect of nursing humanistic care intervention.

**Results:**

Nursing satisfaction: the nursing satisfaction of the experimental group increased from 84.6% to 96.2%, after intervention, satisfaction of the experimental group was 96.2% higher than that of 86.5% of the control group.

**Conclusion:**

Nursing intervention measures based on needs of nursing humanistic care can improve nursing satisfaction, insight and treatment attitude of patients, enhance recovery effect of patients, reduce negative emotions of patients, and benefit recovery of patients' conditions.

## 1. Introduction

Schizophrenia is a serious mental disorder, which is a type of severe mental illness that is caused by dysfunction of the brain under the action of various factors (including biological, psychological, and social factors), resulting in disorders of perception, thinking, emotion, and volitional behavior. It is a mental illness with a high relapse rate and high disability rate, and most of them require lifelong medication [1]. Schizophrenia affects 1% of the world's population worldwide [2], and as of 2010, there were approximately 7.16 million people with schizophrenia in China, accounting for approximately 1/3 of the global total [3]. Patients with schizophrenia are prone to recurrent relapses, and as the disease progresses, patients experience varying degrees of social isolation, disability, and decreased cognitive function and health [4]. The high relapse rate and high disability rate of schizophrenia have now become one of the key public health concerns of the society. The recovery period of schizophrenia refers to the consolidation and maintenance treatment period after schizophrenia patients have been treated systematically with antipsychotic drugs and psychological interventions, and their psychiatric symptoms have been controlled, their self-knowledge has been basically restored, and their condition has been stabilized; although the self-knowledge of patients in this period has been restored, their psychological activities are exceptionally complex and contradictory, and they are extremely prone to negative psychological emotions such as depression and anxiety, which are not conducive to the recovery of their condition, therefore, humanistic care measures for the rehabilitation of schizophrenic patients play an important role in the stability of the overall condition. Rehabilitation not only pursues the stabilization of the condition and the correct perception of the disease, but also includes the patient's emergence from failed interpersonal relationships, complex psychological contradictions, and social discrimination, and rehabilitation is a long process of continuous transformation of goals and directions until the reconstruction of life [5].

The nursing humanistic care cup refers to paying attention to patients' needs and respecting their life values in the nursing process. In addition to providing patients with the necessary diagnostic and technical services, we should also provide spiritual, cultural, emotional, and other multifaceted services to meet patients' physical and mental health needs, which is an interpersonal and loving interaction and fully reflects the concept of people-oriented nursing. The core idea of humanistic care theory is to meet the individual needs of patients, that is, before providing nursing services, we must first accurately understand the different needs of patients with different backgrounds and conditions, so that each patient with different characteristics can receive the most appropriate care and nursing care when they need help. Nursing humanistic care needs are the care and care services that patients need, the nursing help that patients need to achieve a high level of physical, psychological, social, and spiritual harmony in the process of treatment and recovery from their conditions. A nursing humanistic care needs survey is a series of assessments conducted to understand whether and what kind of care patients need in terms of physical, psychological, social, and spiritual care.

Patients in schizophrenia rehabilitation experience long-term closed hospitalization without family members and receive only full-time nursing care from nurses [6], and patients do not have contact with the outside world. This status quo can easily lead to problems such as lack of emotion, information blockage, and lack of communication, and patients in schizophrenia rehabilitation may experience varying degrees of decreased self-care ability and significant social function deficits, so that patients cannot adapt to society after discharge from the hospital. Schizophrenia is mainly treated by long-term oral medication, and although medication can effectively control the positive symptoms of patients, it is difficult to change the negative symptoms such as paucity of thought, emotional indifference, and diminished subjective volitional activity, so effective nursing interventions must be combined with medication in order to achieve a better recovery effect [7]. However, the current traditional caregiving model in psychiatric wards neglects the humanistic care of patients and fails to improve the various aforementioned symptoms left by patients, so it is important to explore the humanistic care of nursing patients in the recovery period of schizophrenia.

Currently, the National Health Planning Commission proposed to strengthen the internal construction of nursing in the “Outline of China's Nursing Career Development Plan 2016–2020” [8], which requires “deepening the ‘patient-centered' service concept, vigorously promoting quality nursing services, and nurses using professional knowledge and skills to provide medical care, observation of illnesses, health Nurses should use their professional knowledge and skills to provide medical care, observation, health guidance, chronic disease management, rehabilitation promotion, psychological care and other services to reflect humanistic care.” World Mental Health Day is celebrated on October 10 every year. The World Health Organization and other organizations hope to raise public awareness of mental health issues around the world through this day, and the Health Planning Commission points out that patients with severe mental disorders are a socially disadvantaged group in great difficulty, with high poverty rates, generally low literacy, low treatment compliance, and a lack of adequate family and social support. In view of these problems, in recent years, the national and local governments have been increasing their support for building the capacity of mental health services and continuously improving the national mental health service system to ensure that people with mental illness enjoy dignity and the integrity that they possess as a person, which shows that the state is paying increasing attention to people with mental illness. Therefore, assessing the current situation of the nursing humanistic care needs of patients recovering from schizophrenia is a concrete manifestation of the equality of patients' lives and the essential attributes of nursing humanistic care, and is an urgent issue to be addressed at the initial stage of implementing nursing humanistic care for patients recovering from schizophrenia.

## 2. Related Work

At present, numerous studies have shown that the implementation of humanistic care model for patients in the recovery period of schizophrenia can effectively improve patients' self-awareness of their mental illness and their compliance with treatment, which can effectively improve their condition and social function and promote their recovery [9]. Studies by foreign scholars point out that implementing humanistic care for patients in the recovery period of schizophrenia to help them improve their living conditions and bad habits, remove adverse psychological factors, and restore their optimal state are the current goals of psychiatric clinical nursing reform [10]. As nursing humanistic care has achieved significant results in nursing practice, the nursing humanistic care needs of patients in schizophrenia recovery and the quality of nurses implementing nursing humanistic care have been continuously emphasized, but some existing studies have shown that at present, due to insufficient allocation of clinical nursing human resources, lack of humanistic education of nursing staff and patients suffering from different degrees of social discrimination, clinical nursing humanistic care practice is rarely implemented from the perspective of nursing humanistic care needs of patients recovering from schizophrenia, and most nursing measures are developed and implemented from the nurse's point of view and less often combined with the patient's point of view [11, 12]. However, existing studies have shown that patients have different levels of need for different nursing humanistic care components [13, 14] and that nursing and patient perspectives on nursing humanistic care needs are not consistent [15]. Therefore, in order to promote patients' recovery and further improve their quality of life, it is worthwhile to investigate the nursing humanistic care needs of patients in schizophrenia recovery from the patient's perspective and how to meet the patients' needs in depth.

Based on the current status of research on nursing humanistic care assessment tools at home and abroad, the research is mainly related to the following aspects, such as the nature of care, care in clinical care, nursing staff and patients' evaluation of caring behavior, caring ability evaluation, caring efficacy evaluation, organizational caring atmosphere evaluation, patients' experience of care, correlation between nursing staff care and patients' satisfaction with nursing services, and care in nursing education. There are 31 types of nursing humanistic care in foreign countries. At present, there are 31 assessment tools related to nursing humanistic care in foreign countries, and most of the domestic scholars use them after Chineseization and improvement. Among the existing assessment tools, fewer can be used to investigate patients' nursing humanistic care needs. (1) The humanistic care assessment tools studied by foreign scholars are commonly used: Care Assessment Questionnaire (CARE ∼ Q), Caring Behavior Assessment Form (CBA), Caring Behavior Inventory (CBI), and Nursing Humanistic Care Inventory (NCI) [16]. (2) The nursing humanistic care needs questionnaires developed by domestic scholars themselves include: a study [17] developed a nursing humanistic care needs questionnaire for inpatients; a study [18] developed a caring behavior evaluation scale for the elderly with the Watson humanistic care theory; and a study [19] developed a nursing humanistic care behavior needs questionnaire with the human hierarchy of needs theory. After searching and reviewing books, they failed to come up with a standard questionnaire for nursing humanistic care needs of patients recovering from schizophrenia [20] pointed out that the only humanistic care literature studies in China are basically Chineseizing foreign scales and using them directly, and truly studying the needs for nursing humanistic care from the perspective of schizophrenia patients, a vulnerable group, and designing the corresponding humanistic care needs assessment This fully illustrates that the theory of nursing care in China is not perfect.

In summary, scholars at home and abroad have made important achievements in nursing humanistic care, but the existing nursing humanistic care needs assessment tools have universal applicability, and there is no nursing humanistic care needs questionnaire for patients recovering from schizophrenia. Therefore, the existing nursing humanistic care needs assessment tools are not suitable for use with patients recovering from schizophrenia. The lack of nursing humanistic care needs assessment tools for patients recovering from schizophrenia has seriously restricted the development of nursing humanistic care and the quality of services for patients recovering from schizophrenia, so the nursing humanistic care needs survey and assessment tools for patients recovering from schizophrenia need to be studied in depth to explore how to develop nursing humanistic care assessment indexes based on the closed management of psychiatric wards in China, combined with the subjective feelings of patients recovering from schizophrenia. This study was carried out in the context of the assessment of the humanistic care needs of patients with schizophrenia. Because of this, this study, from the perspective of nursing humanistic care, combined the actual situation of psychiatric wards and existing tools related to nursing humanistic care assessment, and based on Maslow's hierarchy of needs and Watson's theory of humanistic care, constructed a nursing humanistic care needs survey questionnaire in line with patients recovering from schizophrenia, with the aim of more accurately understanding the current situation of patients' nursing humanistic care needs. The purpose is to develop more effective nursing interventions based on this, aiming to improve the quality of nursing humanistic care for patients recovering from schizophrenia.

## 3. Materials and Methods

### 3.1. Research Objects

From September to December 2021, 110 convalescent patients with schizophrenia in our hospital were selected by convenience sampling method as research objects. The intervention time was 3 months, and data were collected within one week after intervention.

### 3.2. Inclusion Criteria

1. Meeting diagnostic criteria for schizophrenia in the tenth edition of International Classification of Diseases (ICD∼10);
2. The attending psychiatrist diagnosed schizophrenia in the convalescent period, mental symptoms basically disappeared, insight basically recovered, and PANSS score was less than 60;
3. Have complete language comprehension and expression ability;
4. Willing to participate in this research.

### 3.3. Exclusion Criteria

1. Exclude intellectual disability;
2. Serious physical disease.
3. The condition changes beyond the scope of recovery period;
4. The lack of data collection makes it impossible to evaluate the effect.

### 3.4. Falling off Standard

1. The patient is discharged from the hospital;
2. Unwilling to continue to cooperate with research.

### 3.5. Grouping Method

The subjects were randomly numbered from 1 to 110, and random number table method was used to generate random numbers from 1 to 110 using RAND function of Excel software (*n* = 55), and even numbers (*n* = 55) were set as control.

### 3.6. Control

To give psychiatric routine care, the content of psychiatric routine care is as follows:

1. Safe care
2. Daily life care
3. Diet care
4. Sleep care
5. Drug compliance care
6. Visiting nursing

### 3.7. Test

On the basis of routine nursing measures in control, targeted nursing humanistic care needs measures were given.

According to items with relatively high scores of patient needs obtained from the second part of the survey, the corresponding nursing measures that were undertaken are:

1. Psychological care
2. Industrial and recreational nursing
3. Social skills training
4. Life problem solving training
5. Health education
6. Encourage family members to visit
7. Increase social support

### 3.8. Survey Tools

1. General information questionnaire;
2. Questionnaire for nursing satisfaction: 80–100 points are very satisfied; 60–80 points are basically satisfied; less than 60 points are dissatisfied, full score is 100 points, which is evaluated by patients;
3. Insight and Treatment Attitude Questionnaire (ITAQ): it is a half-formulated questionnaire with a total of 11 items. The examination contents include patients' understanding of disease and their attitude toward treatment. All items are scored on a 3-level scale from 0 to 2, with 0 indicating no insight, 1 indicating partial insight, and 2 indicating complete insight. The highest total score of the questionnaire is 22, and the lowest is 0; the higher the total score, the more sufficient the patient's insight. The evaluation physician will evaluate the patient;
4. Inpatient Psychiatric Patient Rehabilitation Outcome Rating Scale (IPROS): to assess daily function of patients, including 5 dimensions (work-therapy situation, living ability, social ability, ability to pay attention to hygiene, concern, and interest), a total of 36 items, each item was scored on a 0–4 scale, with a higher score indicating a worse patient's daily life function;
5. Negative emotions: according to Chinese norm: SDS > 53 points indicate depression, higher scores indicate more severe depression; SAS > 50 points indicate anxiety, and higher scores indicate more severe anxiety.

### 3.9. Evaluation Indicators

1. Nursing satisfaction;
2. Insight and therapeutic attitude;
3. Rehabilitation efficacy;
4. Negative emotions.

### 3.10. Pre-Experiment

Before the start of the formal study, a preliminary experiment was conducted, and 25 patients were selected for a 2-week intervention, in order to discover possible problems in the experimental design, so as to revise intervention plan in time, and also make the research team more familiar with intervention and the procedures and methods to ensure the successful completion of this study.

### 3.11. Quality Control

1. The research participants: they were led by researchers, a clinical nurse intervention was established, and team members were nurses who had worked in psychiatry for more than 2 years and obtained nurse qualification certificates. One month before implementation of intervention, relevant personnel shall be trained according to formulated nursing humanistic care measures every week, and specific methods and precautions shall be explained. Humanitarian care measures are a part of nursing, which can ensure that patients are happy;
2. Research objects: the research objects were selected strictly according to inclusion and exclusion criteria. Before implementing intervention, explain purpose, significance and intervention method of this study to patient, so that patient can fully understand benefit of this intervention, so as to obtain cooperation of patient, and sign informed consent;
3. Data collection: incomplete questionnaires were excluded, and data were checked by double entry.

### 3.12. Statistical Methods

SPSS22.0 statistical software was used for data analysis, *P* < 0.05 indicated statistical significance.

1. The differences in general demographic data of patients were compared by *x*-test;
2. The Mann–Whitney *U* rank sum test was used to compare changes of nursing satisfaction before and after nursing humanistic care intervention;
3. Independent two-sample *t*-test and paired-sample *t*-test were used to compare nursing humanistic care in patients before and after prognosis,
4. The effect of nursing humanistic care intervention in changes of insight, treatment attitude, rehabilitation efficacy, and negative emotion scores were analyzed.

### 3.13. Ethical Principles

1. The principle of informed consent: inform the patient of purpose, significance ,and intervention method of study before implementing intervention. Based on the principle of voluntary participation, the patient has the right to withdraw halfway;
2. Beneficial principle: the nursing measures formulated are based on needed nursing content obtained from patient's investigation, so that the intervention measures are beneficial to the physical and mental health of the patient;
3. Confidentiality principle: an anonymous questionnaire is performed on patients to ensure that no patient-related information is disclosed, and it is only used for this research.

## 4. Results

The exclusion and dropout of patients in this study included a total of 110 rehabilitated patients with CHIZO) Henner, i.e., 55 cases for the experimental and 55 cases for the control group, as detailed in Figure 1.

A total of 110 patients were included in this study, 6 were dropped out, and 104 patients finally completed the study, namely, 52 in experimental and 52 in control. There was no statistical difference in general data such as age, educational level, marital status, hospitalization times, and years of illness of patients, *P* > 0.05, see Figure 2 and Table 1.

Total satisfaction rate % = (very satisfied people + basic satisfied people)/52 × 100%. The rank sum test showed that the total satisfaction rate of patients before intervention was not significant (*P* > 0.05); total satisfaction rate of the experimental group before and after intervention increased from 84.6% to 96.2%. After intervention, the total satisfaction rate of the experimental group was higher than that of control, see Table 2.

As shown in Table 3, the paired *t*-test showed that the insight and treatment attitude scores of patients before the intervention were not significant (*P* > 0.05) and the difference was not statistically significant; the experimental insight and treatment attitude scores before and after the intervention ranged from 8.76 ±2.67 before the intervention to 13.36 ±2.09 after the intervention; after the intervention, the insight and treatment attitude scores of the experimental group were higher than those of the control group.

Two independent samples *t*-test was used to show that there was no statistical significance in evaluation scores of rehabilitation efficacy before intervention, see Table 4.

Using paired *t*-test, it was found that scores of occupational therapy, living ability, social ability, paying attention to hygiene, concern, and interest in the experimental group were increased from 12.36±2.18 points, 9.87±2.65 points, 8.04±1.96 points, and 6.12±1.77 points before intervention. Scores, 9.25±1.69 points decreased to 8.02±1.94 points, 6.51±1.73 points, 5.15±1.06 points, 3.08±0.57 points, and 6.11±1.38 points after intervention. As shown in Table 5, the scores for occupational therapy, life skills, social skills, ability to pay attention to health, concern, and interest in the control group were not statistically significant before and after the intervention (*P* > 0.05).

Two independent samples *t*-test was used to show that after intervention, scores of experimental work situation, living ability, social ability, ability to pay attention to hygiene, concern, and interest were 8.02±1.94 points, 6.51±1.73 points, 5.15±1.06 points, and 3.08±0.57 points, respectively. 11.86±2.54, 9.56±1.68, 7.63±1.04, 5.88±0.49, and 8.73±1.42, all lower than the control (*P* < 0.05), see Table 6.

Two independent samples *t*-test was used to show that negative emotion scores of patients before intervention were not significant (*P* > 0.05), see Table 7.

Using paired *t*-test, it was found that SDS and SAS scores of the experimental group decreased from 55.24±5.91 points and 51.42±5.46 points before intervention to 42.53±4.82 points and 38.45±4.38 points after intervention, all had statistical significance; SDS and SAS scores of the control group had no significance before and after intervention (*P* > 0.05), see Table 8.

Two independent samples *t*-test was used to show that after intervention, SDS score of the experimental group was 42.53±4.8 points and SAS score was 38.45±4.38 points, which were lower than the SDS score of 53.64±5.52 points and SAS score of 48.29±5.37 points in the control group, see Table 9.

## 5. Discussion

With the development of society and improvement of people's quality of life, medical nursing model has undergone corresponding changes. Traditional nursing can no longer meet requirements of patients and their families. The humanities guided by biological-social-psychological modern medical model, nursing management is gradually gaining clinical acceptance. At present, most of the mental hospitals in our country adopt closed nursing mode, ignoring humanistic care and psychological care for patients [21]. Humanistic care nursing is a nursing method that starts from the concept of people-oriented, focuses on patient health, and aims to restore and rebuild social function and healthy behavior of mentally ill patients. It has been widely used in nursing of schizophrenia patients in recent years [22]. The results showed that observation was better than the control group in terms of BPRS measurement, rehabilitation efficacy measurement, and SDSS score. Therefore, humanistic care can effectively improve the level of nursing, improve condition of patients with schizophrenia, promote improvement and recovery of social functions, and improve physical and mental health of patients [23]. It is a nursing management method with good clinical efficacy. Schizophrenia patients are vulnerable in society and should be given adequate humanistic care. Humanistic care nursing is needed for social development, and it is also an embodiment of nursing career progress. In addition, patients should be respected by the government, social, and legal levels, eliminating discrimination, and promoting patients to return to normal work and life as soon as possible, so as to better integrate into society [24]. Humanistic care is beneficial to improve patients' self-confidence, improve their negative emotions, improve their nursing satisfaction, and promote their early integration into society, which is worthy of clinical promotion.

Quality of life is an individual's perception of their place in life, with associated cultural and value systems, involving their physical condition, mental state, degree of independence, social relationships, and their relationship with the environment [25]. Patients with schizophrenia have a lower quality of life than the normal population: patients' cognitive functioning, social dysfunction, social environment, and economic status all influence patients' quality of life; other factors include the severity of symptoms, adverse drug reactions, and patients' attitudes toward medications. Family support for patients also affects patients' quality of life. The SF-36 is a commonly used instrument to measure quality of life [26]. Although it is not specifically designed for quality of life in schizophrenia, it has been used in numerous studies to measure quality of life in schizophrenia [27]. The present study showed that quality of life improved after 12 months of treatment, but the degree of improvement varied, with overall improvements in quality of life being more pronounced and improvements in overall health and emotional functioning greater than medication. This suggests that psychosocial rehabilitation treatment can improve the quality of life of patients with schizophrenia. Studies [28] have reported that classical antipsychotics affect patients' quality of life and that newer antipsychotics are better at improving quality of life in schizophrenia compared to classical antipsychotics and medications. However, a large number of studies have shown that newer antipsychotics have little or no effect on improving quality of life [29]. The impact of psychological interventions on improving patients has been confirmed by a large number of studies with very precise effects [30]. Some studies on psychological interventions for patients with somatic disorders have shown improved quality of life in patients who received psychological interventions [31]. For patients with psychiatric disorders, psychological interventions can also improve their quality of life. A foreign scholar conducted the first study on psychological rehabilitation for patients with schizophrenia and found that their quality of life improved compared to general psychological interventions [32]. All studies have shown that family health education can improve the quality of life of schizophrenia patients [33]. Possible reasons for improving the quality of life in schizophrenia through psychological rehabilitation are health education and family interventions. Preimproving the family atmosphere helps patients to deal with family relationships correctly, corrects incorrect coping strategies and patients' misconceptions about the disease, improves patients' insight, and reduces their sense of stigma. At the same time, psychological rehabilitation reduced patients' negative attitudes toward the disease and symptoms such as anxiety, depression, and fear, and made them more confident in overcoming the disease. Improved adherence also makes medications work better, leading to better clinical outcomes, all of which have a positive effect on quality of life improvement. The nursing staff also benefits through psychological rehabilitation, their level of care and mental health is greatly improved, they are more active and effective in caring for the patient, which contributes to a harmonious family atmosphere where the patient can feel that the family cares for them (her) and reduces the burden on the family.

With the development of society and the improvement of people's quality of life, the medical care model has changed accordingly, and traditional care can no longer meet the requirements of patients and their families. Humanities is guided by the bio-social-psychological modern medical model, and nursing management is gradually gaining clinical recognition. Currently, most psychiatric hospitals in China adopt a closed care model, neglecting humanistic and psychological care for patients. Humanistic care nursing is a nursing approach that focuses on patients' health from a person-centered concept and aims to restore and rebuild the social functions and healthy behaviors of psychiatric patients. In recent years, it has been widely used in the care of patients with schizophrenia [34]. The study [35] found that the observation results were better than the control in terms of BPRS measures, rehabilitation efficacy measures, and SDSS scores. Humanistic care can effectively improve the level of care, improve the condition of schizophrenic patients, promote the improvement and recovery of social function, and improve the physical and mental health of patients, and it is a clinically efficacious method of care management. Patients with schizophrenia are a vulnerable group in society and should be given adequate humanistic care. Humanistic care nursing is a need for social development and a reflection of the progress of nursing. In addition, patients should be respected from governmental, social, and legal levels to eliminate discrimination and facilitate their return to normal work and life as soon as possible so that they can better integrate into society. Humanistic care is conducive to improving patients' self-confidence, improving their negative emotions, increasing their satisfaction with care, and promoting their early integration into society, and is worthy of clinical promotion.

## 6. Conclusion

The overall level of nursing humanistic care needs of patients recovering from schizophrenia was high, and the dimensions of needs were, in descending order, the needs for love and belonging, self-actualization, self-esteem, safety, and physiological needs. The main factors affecting the humanistic care needs of patients in schizophrenia rehabilitation were the number of hospitalizations, years of illness, family attention, and nursing satisfaction, among which the number of hospitalizations and years of illness were positively correlated with patients' needs, and family attention and nursing satisfaction were negatively correlated with patients' needs. In this study, corresponding nursing humanistic care measures were developed and interventions were carried out for patients according to their needs, and the evaluation of intervention effects showed that nursing humanistic care interventions could improve patients' nursing satisfaction, self-knowledge and treatment attitude, rehabilitation efficacy, and reduce patients' negative emotions. Therefore, it is important to implement nursing humanistic care for patients recovering from schizophrenia.

## Figures and Tables

**Figure 1:** The dropout of patients.

**Figure 2:** Schematic diagram of comparison of general information of patients.

**Table 1:** Comparison of general data of patients (*n* = 104).

Project	Classification	Test (*n* = 52)	Control (*n* = 52)	*χ* ^2^	*P* value
Gender	Male	39	40	0.051	0.825
	Female	15	14		

Age (years)	∼31	10	10	0.515	0.917
	32∼46	20	21		
	47∼61	18	17		
	Over 61 years old	8	5		

Educational level	Elementary school and below	12	11	0.209	0.993
	Junior high school	25	24		
	High school or secondary school	12	13		
	College	7	6		
	Undergraduate and above	3	3		

Marital status	Unmarried	12	11	0.655	0.723
	Married	20	23		
	Widowhood/Divorce	25	22		

Primary caregiver	Parent	10	8	0.818	0.938
	Children	15	16		
	Spouse	15	17		
	Brothers and sisters	10	7		
	Other	5	5		

Number of hospitalizations	1 time	9	11	0.412	0.816
	2 times	13	14		
	3 times or more	34	30		

Years of illness	Within 1 year	7	9	0.481	0.785
	1∼3 years	19	20		
	Over 3 years	27	25		

Monthly household income (yuan)	Below 2000	11	9	0.531	0.764
	2000∼5000	27	25		
	More than 5000	13	16		

Family attention	Difference	9	8	0.163	0.921
	Generally	25	27		
	Better	19	17		

Nursing satisfaction	Dissatisfied	10	9	0.088	0.956
	Basically satisfied	24	24		
	Very satisfied	20	19		

**Table 2:** Comparison of nursing satisfaction of patients before and after intervention.

Group	Before intervention				After intervention				U	*P*
	Very satisfied	Basically satisfied	Dissatisfied	Total satisfaction rate (%)	Very satisfied	Basically satisfied	Dissatisfied	Total satisfaction rate (%)		
Test (*n* = 52)	20	26	9	84.5	38	15	3	96.3	857.1	0.001
Control (*n* = 52)	19	26	10	82.9	19	36	8	86.6	1318.1	0.809

*U*	1313.6				839.4					
*P*	0.786				0.001					

**Table 3:** Comparison of insight and treatment attitude before and after intervention ($\bar{X}\pm S$).

Group	Before intervention	After intervention	*t*	*P*
Test (*n* = 52)	8.76 ± 2.67	13.36 ± 2.09	−9.85	0.001
Control (*n* = 52)	8.65 ± 2.16	9.39 ± 2.02	−1.737	0.081
*t*	0.169	10.022		
*p*	0.866	0.001		

**Table 4:** Comparison of rehabilitation efficacy evaluation scores of patients before intervention ($\bar{X}\pm S$).

Group	Occupational therapy	Living ability	Social skills	Pay attention to hygiene ability	Care and interest
Test (*n* = 52)	12.34±2.20	9.88±2.64	8.06±1.94	6.14±1.75	9.27±1.67
Control (*n* = 52)	12.81±2.90	10.16±2.46	7.83±1.74	6.01±0.58	8.91±1.52
*t*	−0.937	−0.555	0.526	0.350	1.051
*p*	0.351	0.577	0.601	0.726	0.295

**Table 5:** Comparison of rehabilitation efficacy evaluation scores before and after intervention ($\bar{X}\pm \text{S}$).

Group	Test (*n* = 52)		*t*	*p*	Control (*n* = 52)		*t*	*p*
	Before intervention	After intervention			Before intervention	After intervention		
Occupational therapy	12.35±2.19	8.04±1.92	10.721	0.001	12.81±2.89	11.85±2.55	1.823	0.072
Living ability	9.88±2.64	6.52±1.71	7.653	0.001	10.14±2.46	9.55±1.67	1.422	0.157
Social skills	8.06±1.95	5.17±1.04	9.353	0.001	7.84±1.73	7.65±1.02	0.788	0.432
Pay attention to hygiene ability	6.14±1.75	3.07±0.57	11.789	0.001	6.05±0.54	5.89±0.50	1.455	0.147
Care and interest	9.23±1.71	6.13±1.36	10.376	0.001	8.94±1.49	8.75±1.41	0.661	0.511

**Table 6:** Comparison of rehabilitation efficacy evaluation scores of patients after intervention ($\bar{X}\pm S$).

Group	Occupational therapy	Living ability	Social skills	Pay attention to hygiene ability	Care and interest
Test (*n* = 52)	11.85±2.55	9.57±1.67	7.61±1.06	5.86±0.51	8.75±1.40
Control (*n* = 52)	8.03±1.95	6.52±1.72	5.13±1.08	3.06±0.58	6.12±1.37
*t*	8.665	9.121	12.041	26.862	9.540
*P*	0.001	0.001	0.001	0.001	0.001

**Table 7:** Comparison of negative emotions before intervention ($\bar{X}\pm S$).

Group	SDS	SAS
Test (*n* = 52)	55.25±5.92	51.43±5.45
Control (*n* = 52)	54.88±5.73	50.02±5.52
*T*	0.325	1.293
*P*	0.745	0.197

**Table 8:** Comparison of negative emotions before and after intervention ($\bar{X}\pm S$).

Group	Test (*n* = 52)		*t*	*p*	Control (*n* = 52)		*t*	*p*
	Before intervention	After intervention			Before intervention	After intervention		
SDS	55.25±5.90	42.51±4.84	12.017	0.001	54.88±5.75	53.65±5.51	1.112	0.265
SAS	51.43±5.45	38.47±4.36	13.362	0.001	50.01±5.53	48.27±5.35	1.631	0.105

**Table 9:** Comparison of negative emotions after intervention ($\bar{X}\pm S$).

Group	SDS	SAS
Test (*n* = 52)	53.66±5.50	48.27±5.39
Control (*n* = 52)	42.55±4.80	38.44±4.39
*T*	10.931	10.238
*P*	0.001	0.001

## Data Availability

The experimental data used to support the findings of this study are available from the corresponding author upon request.

## References

[1] Naomi G., Kwadwo Wisdom M., Mensah I., Collins Kwabena B., Anderson Mensah P., Badu E. (2022). For me I see MINE to be a family sickness–consumers understanding and perception of the etiology of mental illness in community-based residential facilities in Ghana. *Mental Health, Religion & Culture*.

[2] Özdemir A. A., Kavak Budak F. (2022). The effects of mindfulness-based stress reduction training on hope, psychological well-being, and functional recovery in patients with schizophrenia. *Clinical Nursing Research*.

[3] Goman C., Patterson C., Moxham L., Harada T., Tapsell A. (2020). Alternative mental health clinical placements: knowledge transfer and benefits for nursing practice outside mental healthcare settings. *Journal of Clinical Nursing*.

[4] Solomon B., Sutton D., McKenna B. (2021). The experience and meaning of recovery‐oriented practice for nurses working in acute mental health services. *International Journal of Mental Health Nursing*.

[5] Damsgaard J. B., Angel S. (2021). Living a meaningful life while struggling with mental health: challenging aspects regarding personal recovery encountered in the mental health system. *International Journal of Environmental Research and Public Health*.

[6] Tasijawa F. A., Suryani S., Sutini T., Maelissa S. R. (2021). Recovery from ‘schizophrenia’: perspectives of mental health nurses in the Eastern island of Indonesia. *Belitung Nursing Journal*.

[7] Salzmann-Erikson M., Sjödin M. (2018). A narrative meta-synthesis of how people with schizophrenia experience facilitators and barriers in using antipsychotic medication: implications for healthcare professionals. *International Journal of Nursing Studies*.

[8] Harris B. A., Panozzo G. (2019). Therapeutic alliance, relationship building, and communication strategies-for the schizophrenia population: an integrative review. *Archives of Psychiatric Nursing*.

[9] Bellier-Teichmann T., Antonini M., Delmas P. (2022). Assessing resources in a population of hemodialysis patients: a new approach to improve quality of care. *Journal of Contemporary Psychotherapy*.

[10] Neathery M., Taylor E. J., He Z. (2020). Perceived barriers to providing spiritual care among psychiatric mental health nurses. *Archives of Psychiatric Nursing*.

[11] Fiorillo A., Barlati S., Bellomo A. (2020). The role of shared decision-making in improving adherence to pharmacological treatments in patients with schizophrenia: a clinical review. *Annals of General Psychiatry*.

[12] Cripps L., Deyell Hood C. (2020). Recovery and mental health: exploring the basic characteristics of living well with mental illness. *Therapeutic Recreation Journal*.

[13] Masedo A., Grandón P., Saldivia S. (2021). A multicentric study on stigma towards people with mental illness in health sciences students. *BMC Medical Education*.

[14] Loh S. Y. (2018). Interdisciplinary rehabilitation to facilitate recovery of people living with long-term schizophrenia in developing countries. *Psychotic Disorders: Update*.

[15] Hortal‐Mas R., Moreno‐Poyato A. R., Granel‐Giménez N. (2022). Sexuality in people living with a serious mental illness: a meta‐synthesis of qualitative evidence. *Journal of Psychiatric and Mental Health Nursing*.

[16] Nasrollah S., Rafii F., Ghezeljeh T. (2019). Discriminative nursing care: a grounded theory study. *Journal of Family Medicine and Primary Care*.

[17] O’Keeffe D., Sheridan A., Kelly A. (2018). ‘Recovery’in the real world: service user experiences of mental health service use and recommendations for change 20 years on from a first episode psychosis. *Administration and Policy in Mental Health and Mental Health Services Research*.

[18] Eiroa-Orosa F. J., Garcia-Mieres H. (2019). A systematic review and meta-analysis of recovery educational interventions for mental health professionals. *Administration and Policy in Mental Health and Mental Health Services Research*.

[19] Pratt H., Moroney T., Middleton R. (2021). The influence of engaging authentically on nurse–patient relationships: a scoping review. *Nursing Inquiry*.

[20] Lysaker P. H., Dimaggio G., Hamm J. A., Leonhardt B. L., Hochheiser J., Lysaker J. T. (2019). Disturbances in self-experience in schizophrenia: metacognition and the development of an integrative recovery-oriented individual psychotherapy. *Psychopathology*.

[21] Douglas L., Donohue G., Morrissey J. (2022). Patient experience of physical restraint in the acute setting: a systematic review of the qualitative research evidence. *Issues in Mental Health Nursing*.

[22] Ramon S. (2018). The place of social recovery in mental health and related services. *International Journal of Environmental Research and Public Health*.

[23] Jackson-Blott D. K., Hare D. D., Morgan D. S., Davies D. B. (2019). Recovery from psychosis in a forensic service: assessing staff and service users’ perspectives using Q methodology. *Journal of Forensic Psychology Research and Practice*.

[24] Craig T. J. (2019). Social care: an essential aspect of mental health rehabilitation services. *Epidemiology and Psychiatric Sciences*.

[25] Forde R., Peters S., Wittkowski A. (2020). Recovery from postpartum psychosis: a systematic review and metasynthesis of women’s and families’ experiences. *Archives of Women’s Mental Health*.

[26] Rossi R., Socci V., Rossi A. (2022). Personal recovery in Schizophrenia: a narrative review. *Recovery and Major Mental Disorders*.

[27] Isaacs A. N., Brooks H., Lawn S., Mohammadi L., Vicary E., Sutton K. (2022). Effectiveness of personal recovery facilitators in adults with schizophrenia and other psychoses: a systematic review of reviews and narrative synthesis. *Schizophrenia Research*.

[28] Mallet J., Le Strat Y., Dubertret C., Gorwood P. (2022). Recovery-oriented psychopharmacological interventions in schizophrenia. *Recovery and Major Mental Disorders*.

[29] Suryani S., Hidayah N., Sutini T., Al-Kofahy L. (2022). The Indonesian survivors’ perspective about recovery from schizophrenia: an exploratory study. *Jurnal Keperawatan Padjadjaran*.

[30] Goodsmith N., Cohen A. N., Pedersen E. R., Evans E., Young A. S., Hamilton A. B. (2022). Predictors of functioning and recovery among men and women veterans with schizophrenia. *Community Mental Health Journal*.

[31] Jongkind A., Hendriks M., Grootens K., Beekman A. T. F., van Meijel B. (2022). Evaluation of a collaborative care program for patients with treatment-resistant schizophrenia: protocol for a multiple case study. *JMIR Research Protocols*.

[32] Gowda G. S., Isaac M. K. (2022). Models of care of schizophrenia in the community—an international perspective. *Current Psychiatry Reports*.

[33] Caqueo-Urízar A., Ponce-Correa F., Urzúa A. (2022). Effects of recovery measures on internalized stigma in patients diagnosed with schizophrenia. *International Journal of Mental Health and Addiction*.

[34] Tirupati S., Padmavati R., Kumar S., Mohanraj R. (2022). Cross-cultural study of recovery in people with schizophrenia: methodology. *Journal of Psychosocial Rehabilitation and Mental Health*.

[35] Sims S., Hepsipa Omega Juliet S., Joseph J. (2022). Acceptability of peer support for people with schizophrenia in Chennai, India: a cross sectional study amongst people with lived experience, caregivers, and mental health professionals. *Frontiers in Psychiatry*.

